RETRACTED

# LncRNA NEAT1/miR‐185‐5p/IGF2 axis regulates the invasion and migration of colon cancer

**DOI:** 10.1002/mgg3.1125

**Published:** 2020-02-20

**Authors:** Shu‐tong Zhuang, Yan‐juan Cai, Hong‐peng Liu, Ying Qin, Jian‐feng Wen

**Affiliations:** ^1^ Department of Gastrointestinal Surgery Health Science Center The First Affiliated Hospital of Shenzhen University Shenzhen Guangdong China; ^2^ Shenzhen Second People's Hospital Shenzhen Guangdong China; ^3^ Health Science Center The First Affiliated Hospital of Shenzhen University Shenzhen Guangdong China

**Keywords:** colon cancer, IGF2, LncRNA NEAT1, miR‐185‐5p

## Abstract

**Background:**

Long noncoding RNAs (lncRNA) are important in the growth and metastasis of colon cancer. The objective of this study was to describe the potential role of lncRNA *NEAT1* in the progression of colon cancer.

**Methods:**

Quantitative real‐time polymerase chain reaction was used for detecting *NEAT1*, miR‐185‐5p, and *IGF2* in colon cancer cells and tissues. The potential diagnostic value of *NEAT1* in colon cancer was analyzed with the receiver operating characteristic curve. Kaplan–Meier method was applied for evaluating the association between *NEAT1* expression and the overall survival of osteosarcoma patients, whereas Transwell assay was introduced to examine the potential invasion and migration of colon cancer cells. In addition, the binding of *NEAT1*/*IGF2* to miR‐185‐5p was confirmed by RNA pull‐down and RNA‐binding protein immunoprecipitation assays and dual‐luciferase reporter gene assay. Finally, rescue experiments were conducted to confirm the role of *NEAT1*/miR‐185‐5p/*IGF2* axis in colon cancer.

**Results:**

Colon cancer patients with low *NEAT1* expression presented with longer overall survival than those with high expression. The migration and invasion of colon cancer cells were considerably promoted by overexpressed *NEAT1*. Both *NEAT1* and *IGF2* bound to miR‐185‐5p.

**Conclusion:**

*NEAT1* upregulate *IGF2* expression through absorbing miR‐185‐5p to enhances the migration and invasion of colon cancer cells.

## Graphical abstract

Increasing evidence suggest that long noncoding RNAs (lncRNA) expression alterations have a vital impact in the process of biological process in cancer. However, the role of lncRNAs in colorectal cancer remains largely to be explored. Here we reported that NEAT1 upregulate IGF2 expression through absorbing miR‐185‐5p to enhances the migration and invasion of colon cancer cells.

## 1 INTRODUCTION

Colon cancer ranks the third and fourth highest prevalence and mortality in cancers worldwide, respectively (Zeng, Zhu, Li, & Kang, 2017). Over one million colon cancer cases newly emerge, and approximate 700,000 individuals die of this cancer each year (Haggar & Boushey, 2009). Colon cancer is high in the 40–50 age group (Zhai, Xue, Liu, Guo, & Chen, 2017). The occurrence and development of colon cancer involve multiple factors, including inactivated tumor suppressor genes and activated oncogenes (Fearon & Vogelstein, 1990). Surgery is the primary therapy for colon cancer and patients exhibit a 5‐year survival rate of 50% following surgery (Shi et al., 2014). However, 15%–20% patients experience recurrence following treatment. Tumor recurrence following curative surgery is a major hindrance for the improvement of overall survival (Gerger et al., 2011). Therefore, to improve the clinical outcome of colon cancer, the exploration of its pathogenesis becomes necessary.

RETRACTED

As a noncoding RNA with over 200 nucleotides in length, long noncoding RNAs (lncRNA) cannot encode proteins as a result of the absence of open reading frame (Yu, Nangia‐Makker, Farhana, & Majumdar, 2017). LncRNA has long been recognized as the noise of genomic transcription free of biological role. However, lncRNA has been shown to both directly regulate gene expression and interact with miRNA as a ceRNA (competing endogenous RNA) from recent studies (Zhang et al., 2016). The potential role of lncRNA in the regulation of malignant manifestations of tumor cells has attracted extensive attentions (Tay, Rinn, & Pandolfi, 2014; Zhou et al., 2016). Multiple tumors (e.g., prostate cancer, esophageal cancer, cervical cancer, cholangiocarcinoma) have showed abnormal expression of lncRNAs (Dong et al., 2017; Liu et al., 2017; Peng, Yuan, Jiang, Tang, & Li, 2016; Wang et al., 2016). In spite of some advances, there is few studies on lncRNA in colon cancer.

Previous studies have shown high expression of lncRNA *NEAT1* in hepatocellular carcinoma, which is strongly associated with the recurrence, portal vein tumor thrombus, and tumor size. *NEAT1* is considered as an independent prognostic factor for hepatocellular carcinoma from multivariate analysis (Wang, Zou, Song, & Chen, 2017; Zheng et al., 2018). In vitro experiments have demonstrated that long noncoding RNA *NEAT1* contributes to laryngeal squamous cell cancer by the regulation of miR‐107/CDK6 pathway (Wang et al., 2016). Rare reports exist on the clinical significance of lncRNA *NEAT1* in colon cancer. This study investigated the specific expression mode of *NEAT1* and described its biological roles in the development of colon cancer.

## 2 MATERIALS AND METHODS

### 2.1 Ethical compliance

The study obtained the approval opinion from the Ethics Committee of Shenzhen Second People's Hospital.

### 2.2 Tissue samples

Samples were collected according to the agreement of the Medical Ethics Committee of Shenzhen Second People's Hospital. All patients provided the informed consent. This study enrolled 10 colon cancer patients who underwent surgery in Shenzhen Second People's Hospital from January 2017 to December 2018. Tissue samples were maintained in liquid nitrogen before RNA extraction. Among all patients enrolled, no antitumor treatment was received before operation, such as surgery, chemotherapy, and radiotherapy.

RETRACTED

### 2.3 Cell culture and transfection

American Type Culture Collection (ATCC) provided colon cancer cell lines (SW620 HT‐29, HCT 116, LoVo, and SW480) and normal colon epithelial cells (NCM460). Culture medium was Roswell Park Memorial Institute 1640 (HyClone) containing 10% fetal bovine serum (FBS) (Gibco), 100 μg/ml streptomycin, and 100 μg/ml penicillin. Cells were cultured in a 5% CO_2_ incubator at 37°C.

Cell transfection was done using Lipofectamine 2000 (Invitrogen) at 70%–80% of confluence. In brief, small interference RNA or pcDNA was subject to dilution in Opti‐MEM, and followed by mixing with RNA/DNA‐Lipofectamine 2000 after 5 min. Transfection solution was used in each well after 20 min. At 48 hr, transfected cells were harvested for subsequent experiments.

### 2.4 Quantitative real‐time polymerase chain reaction

TRIzol reagent (Invitrogen) was applied for extracting total RNA. MicroRNAs were isolated using the two‐column protocol of the High Pure miRNA Isolation Kit (Sigma‐Aldrich) resulted enriched miRNA fraction. In brief, Binding Buffer was used to produce supernatant of centrifuge lysate from colon cancer tissues or cell lines. Then, the purified small RNA was isolated according to the two‐column protocol of manufacturer's instructions. Then, Primescript RT Reagent (TaKaRa) was used for synthesizing their relative complementary deoxyribose nucleic acid. Quantitative real‐time polymerase chain reaction (qRT‐PCR) was done using SYBR® Premix Ex Taq™ Reagent (TaKaRa) and StepOne Plus Real‐Time PCR system (Applied Biosystems) at 95 °C, 95 °C, 58 °C, and 74 °C for 5 min, 15, 30, and for 30 s, respectively, in a total of 40 cycles. *GAPDH* was used as an endogenous control for lncRNA and mRNA. The expression of miRNA was normalized to small nuclear *U6*. The 2^−ΔΔCt^ method was applied to quantify gene expression. The following primers were applied for qRT‐PCR:

*GAPDH*, F: GCACCGTCAAGGCTGAGAAC, R: GGATCTCGCTCCTGGAAGATG

*U6*, F: CTCGCTTCGGCAGCACA, R: AACGCTTCACGAATTTGCGT

*NEAT1*, F: CTTCCTCCCTTTAACTTATCCATTCAC, R: CTCTTCCTCCACCATTACCAACAATAC; *IGF2*, F: GTGGCATCGTTGAGGAGTG, R: CACGTCCCTCTCGGACTTG; miR‐185‐5p, F: ACACTCCAGCTGGGAGUCCUUGACGGAAAG, R: CTCAACTGGTGTCGTGGAGTCGGCAATTCAGTTGAGUCUCUCCA.

RETRACTED

### 2.5 Western blot

Total proteins were gained after cells were lysed in RIPA buffer (Beyotime) for 30 min and were then centrifuged at 17,000 *g* at 4°C for 45 min. Protein concentrations were determined by BCA protein assay kit (Beyotime). Protein samples were subjected to SDS‐PAGE and electrophoretically transferred to PVDF membranes (Millipore). After blocking in 5% nonfat milk at room temperature for 2 hr, membranes were then incubated with primary antibodies as follows: IGF2 (1:100, ab170304, Abcam), vimentin (1:1000, ab92547, Abcam), cytokeratin 19 (1:1000, ab52625, Abcam), E‐cadherin (1:500, ab15148, Abcam), and GAPDH (1:1000, sc‐25778). After washed three times with TBST, membranes were incubated with horseradish peroxidase conjugated secondary antibodies at room temperature for 2 hr. Immunoblots were visualized with ECL (enhanced chemiluminescence) Kit (Beyotime) and scanned using ChemImager 5500 V2.03 software (Alpha Innotech).

### 2.6 Transwell cell invasion and migration assay

With cells suspended in 1.0 × 10^5^/ml serum‐free medium, Matrigel precoated Transwell chamber or that without precoating was placed in 24‐well plates. The apical chamber contained 200 μl suspension and the basolateral chamber had 500 μl medium containing 10% FBS. At 48 hr, chambers were removed and penetrating cells were fixated in 5% paraformaldehyde for 20 min and stained with 0.1% crystal violet for 20 min. Penetrating cells of each sample were collected from four random fields for counting (magnification 20×). Matrigel was used for precoating Transwell chambers for invasion assay.

### 2.7 Subcellular fractionation location

The location of *NEAT1* in colon cancer cells was determined using a PARIS Kit (Life Technologies) according to the manufacturer's instructions, and fractions of the nucleus and cytoplasm were isolated. RNAs were diluted and tested via qRT‐PCR to analyze *NEAT1*, GAPDH, and U6 expression levels with GAPDH as the cytoplasmic control and U6 as the nuclear control.

### 2.8 RNA pull‐down assay

Colon cancer cells were transiently transfected with biotinylated lncRNA‐*NEAT1* WT, lncRNA‐*NEAT1* MUT, and negative control (JINKAIRUI), respectively, and then harvested. Cell lysates were incubated with Dynabeads/M280 Streptavidin (Invitrogen) according to the manufacturer's protocol. Similarly, the synthesized biotinylated DNA probe complementary to *NEAT1* was incubated with Dynabeads/M280 Streptavidin (Invitrogen) to generate probe‐coated beads. Then, cell lysates were incubated with the probe‐coated beads at 4°C overnight. The RNA complexes bound to these beads were eluted and detected by qRT‐PCR analysis.

RETRACTED

### 2.9 RNA‐binding protein immunoprecipitation assay

RNA‐binding protein immunoprecipitation (RIP) assay was performed using Magna RIP™ RNA‐binding protein immunoprecipitation kit (Millipore) according to the manufacturer's guidelines with minor modifications. Briefly, the magnetic beads were incubated with 5 μg anti‐AGO2 (ab32381, Abcam) or anti‐IgG antibodies for 30min at room temperature to generate antibody‐coated beads. Colon cancer cells (1 × 10^7^) were lysed in 100 μl RIP lysis buffer and then diluted with 900 μl RIP immunoprecipitation buffer and incubated with the antibody‐coated beads overnight at 4°C. After that, beads were washed six times using RIP wash buffer. The immunoprecipitate was treated with Proteinase K at 55°C for 30 min. And the isolated RNA was extracted using TRIzol regent (Invitrogen), followed by qRT‐PCR.

### 2.10 Dual‐luciferase reporter gene assay

We inserted the binding site of *NEAT1* and *IGF2* into the KpnI and SacI sites of pGL3 promoter vector (Realgene) to construct the following fragments: pGL3‐*NEAT1*‐Wild, pGL3‐*NEAT1*‐Mut, pGL3‐*IGF2*‐Wild, and pGL3‐*IGF2*‐Mut. Cells were plated into 24‐well plates and cultured to 50%–70% density. Then we cotransfected 80 ng plasmid, 5 ng renilla luciferase vector pRL‐SV40, 50 nM miR‐185‐5p mimics and negative control into cells using lipofectamine 2000 (Invitrogen). After incubation for 48 hr, changes in luciferase activity were analyzed through the dual Glo luciferase assay system (Promega) in accordance with the manufacturer's protocol. All above experiments were done in triplicate.

### 2.11 Statistical analyses

All statistical analyses were performed with SAS9.1 Software (SAS Institute Inc.). Data were reported as mean ± *SD*. Measurement data in homogeneity of variance and normal distribution were analyzed by *t* test. The potential diagnostic value of *NEAT1* in colon cancer was evaluated by the receiver operating characteristic (ROC) curve, whereas the survival of colon cancer patients was analyzed with Kaplan–Meier method. *p* < .05 was accepted as statistical difference.

## 3 RESULTS

### 3.1 Highly expressed *NEAT1* in colon cancer

Quantitative real‐time polymerase chain reaction was used for examining the expression levels of miR‐185‐5p, *IGF2,* and *NEAT1* in 10 colon cancer tissues and matched normal tissues, and showed a high expression of *NEAT1* and *IGF2* and a low expression of miR‐185‐5p in colon cancer tissues relative to the controls (Figure 1a–d). Colon cancer patients were stratified into low‐level and high‐level groups by the median *NEAT1* expression. Survival analysis indicated that the overall survival of colon cancer patients in high‐level group was less than those in low‐level group (Figure 1e). It is worth mentioning that, there are two isoforms of *NEAT1*, named *NEAT1_1* and *NEAT1_2,* respectively. Here, we focused on the long isoform (*NEAT1_2*) for its higher abundance in colon cancer cell lines (Figure S1a). Moreover, based on ROC curve, *NEAT1* was shown to be of diagnostic potential for distinguishing colon cancer tissues from normal ones (AUC = 0.89, Figure 1f). It turned out that an abnormal expression of *NEAT1*, *IGF2,* and miR‐185‐5p may be crucial in the development of colon cancer.

RETRACTED

**Figure 1:** Highly expressed *NEAT1* in colon cancer. (a) High *NEAT1* expression in colon cancer tissues relative to the controls by QRT‐PCR. (b) Low miR‐185‐5p expression in colon cancer tissues relative to the controls by QRT‐PCR. (c and d) High *IGF2* expression in colon cancer tissues relative to the controls by both QRT‐PCR and Western blot. (e) Shorter overall survival of colon cancer patients in high‐level group than those in low‐level group by survival analysis. (f) Potential diagnostic value of *NEAT1* for distinguishing colon cancer tissues from normal ones as confirmed by ROC curve (AUC = 0.89). qRT‐PCR, quantitative real‐time polymerase chain reaction; ROC, receiver operating characteristic. **p < .01, ***p < .001

### 3.2 Overexpressed *NEAT1* promoted invasion and migration of colon cancer cells

Like the expression in colon cancer tissues, a high *NEAT1* expression was observed in colon cancer cell lines (SW620, HT‐29, HCT 116, LoVo, and SW480) than normal colon epithelial cells (NCM460). Among these two cells that were applied for subsequent experiments, SW480 cells showed a relatively high expression of *NEAT1*, whereas HT‐29 cells showed a low expression (Figure 2a). For the assessment of biological roles of *NEAT1*, *NEAT1* expression in SW480 and HT‐29 cells was downregulated and upregulated by transfecting with si‐*NEAT1* and pcDNA‐*NEAT1*, respectively (Figure 2b,c). Overexpressed *NEAT1* in HT‐29 cells contributed to the invasion and migration as showed by Transwell migration and invasion assays. On the contrary, *NEAT1* knockdown showed inhibiting effect on their invasion and migration in SW480 (Figure 2d). In this study, EMT‐related genes in colon cancer cells were determined. Overexpressed *NEAT1* in HT‐29 cells showed upregulation of vimentin and downregulation of cytokeratin 19 and E‐cadherin (Figure 2e). Inversely, downregulation of vimentin and upregulation of cytokeratin 19 and E‐cadherin were observed in SW480 cells with *NEAT1* knockdown (Figure 2f).

**Figure 2:** Overexpressed *NEAT1* promoted the migration and invasion of colon cancer cells. (a) High *NEAT1* expression was observed in colon cancer cell lines (SW620, HT‐29, HCT 116, LoVo, and SW480) relative to normal colon epithelial cells (NCM460). (b) *NEAT1* expression was considerably upregulated by transfecting of pcDNA‐*NEAT1* in HT‐29 cells. (c) *NEAT1* expression was considerably downregulated by transfecting of si‐*NEAT1* in SW480 cells. (d) Transfection of pcDNA‐*NEAT1* in HT‐29 cells considerably contributed to the migration and invasion, whereas transfection of si‐*NEAT1* in SW480 cells considerably suppressed the migration and invasion. (e and f) Western blot analysis showed that transfection with pcDNA‐*NEAT1* in HT‐29 cells upregulated vimentin, but downregulated cytokeratin 19 and E‐cadherin. Transfection with si‐*NEAT1* in SW480 cells presented with the contrary trends. *p < .05

RETRACTED

### 3.3 *NEAT1* upregulated *IGF2* expression

In previous studies, ceRNA has been considered important to exert the biological role of lncRNA (Gu, Li, Jin, Liu, & Wei, 2017; Yu, Zhao, et al., 2017). Thus, through bioinformatics, it was predicted that both *NEAT1* and *IGF2* presented with binding sites for miR‐185‐5p. Colon cancer cells showed higher *IGF2* expression compared with NCM460 cells (Figure 3a). *IGF2* expression was considerably upregulated or downregulated at protein and mRNA levels, respectively, through transfection of pcDNA‐*IGF2* in HT‐29 cells or si‐*IGF2* in SW480 cells (Figure 3b,d). *IGF2* expression was positively regulated by *NEAT1* as demonstrated by subsequent qRT‐PCR data (Figure 3c). Western blot analysis also yielded similar association at their protein levels (Figure 3e).

**Figure 3:** *NEAT1* upregulated *IGF2* expression. (a) HT‐29 and SW480 cells showed higher *IGF2* expression than NCM460 cells. (b and d) The mRNA and protein levels of *IGF2* expression were considerably upregulated by transfecting of pcDNA‐*IGF2* in HT‐29 cells. The mRNA and protein levels of *IGF2* expression were considerably downregulated by transfecting of si‐*IGF2* in SW480 cells. (c, e) The mRNA and protein levels of *IGF2* expression were upregulated by transfecting of pcDNA‐*NEAT1* in HT‐29 cells. The mRNA and protein levels of *IGF2* expression were downregulated by transfecting of si‐*NEAT1* in SW480 cells. *p < .05

### 3.4 *NEAT1* could bind to *IGF2* and miR‐185‐5p

Long noncoding RNAs function in a manner depending on their subcellular distribution. Hence, qRT‐PCR was adopted to examine *NEAT1* expression in the nucleus and cytoplasm of colon cancer cells. *NEAT1* was primarily present in the cytoplasm of colon cancer cells (Figure S1b). So, *NEAT1* may participate in the development of colon cancer through posttranscriptional regulation. Given that *NEAT1* may participate in the development of colon cancer through posttranscriptional regulation, it was assumed to act as a ceRNA in the development of colon cancer. According to bioinformatics prediction (http://starbase.sysu.edu.cn), the binding sites between miR‐185‐5p and NEAT1 in the binding region (chr11: 65443172–65443195) is similar to the binding sites between miR‐185‐5p and IGF2. Based on qRT‐PCR data, MiR‐185‐5p was lowly expressed in colon cancer cells relative to NCM460 cells (Figure 4a). Through plasmid transfection, miR‐185‐5p mimics or inhibitor considerately downregulated and upregulated miR‐185‐5p expression in SW480 and HT‐29 cells, respectively (Figure 4b). The construction of Luciferase reporter plasmids (*NEAT1*‐WT, *NEAT1*‐MUT, *IGF2*‐WT, *IGF2*‐MUT) was performed on the basis of the predicted binding sites to miR‐185‐5p (Figure 4c). The data indicated that luciferase activity was inhibited in colon cancer cells after cotransfection with miR‐185‐5p mimics and *NEAT1*‐WT/*IGF2*‐WT, suggesting that *NEAT1* and *IGF2* bound to miR‐185‐5p (Figure 4d). In addition, as the outcomes of a RIP‐binding assay presented, the level of *NEAT1* and miR‐185‐5p was higher in anti‐Ago2 group than that in antinormal IgG group which indicating that *NEAT1* and miR‐185‐5p were in the same RNA induced silencing complex (Figure 4e). The specific interaction between miR‐185‐5p and *NEAT1* was further demonstrated by RNA pull‐down assay using biotin‐labeled *NEAT1*. miR‐185‐5p was pulled down by *NEAT1*, whereas *NEAT1* mutant with disrupting putative‐binding sequence resulted in failure of miR‐185‐5p coprecipitation. These results validated that the recognition of miR‐185‐5p to *NEAT1* was in a sequence‐specific manner (Figure 4f). Furthermore, Western blot revealed negative regulation of miR‐185‐5p on *IGF2* expression (Figure 4g).

RETRACTED

**Figure 4:** *IGF2* and *NEAT1* could bind to miR‐185‐5p. (a) NCM460 cells showed high expression of MiR‐185‐5p relative to HT‐29 and SW480 cells. (b) The miR‐185‐5p expression in SW480 or HT‐29 cells was considerably downregulated or upregulated by transfecting of miR‐185‐5p mimics or inhibitor, respectively. (c) Potential‐binding sites of *NEAT1* and *IGF2* to miR‐185‐5p. (d) *NEAT1* and *IGF2* could bind to miR‐185‐5p by dual‐luciferase reporter gene assay. (e) *NEAT1* could bind to miR‐185‐5p by RIP assay. (f) *NEAT1* could bind to miR‐185‐5p as further proved by RNA pull‐down assay. (g) Transfection of miR‐185‐5p mimics in HT‐29 cells downregulated *IGF2* expression, whereas transfection of miR‐185‐5p inhibitor iSW480 upregulated protein levels of *IGF2* expression. RIP, RNA‐binding protein immunoprecipitation. *p < .05

### 3.5 *NEAT1*/MiR‐185‐5p axis was important in migratory and invasive potentials of colon cancer

Finally, the effect of miR‐185‐5p/*NEAT1* on cellular performances of colon cancer was evaluated. HT‐29 cells with overexpressed *IGF2* contributed to migratory and invasive potentials, whereas SW480 cells with *IGF2* knockdown presented with the contrary trends (Figure 5a). It may be concluded the promotive role of *IGF2* on migratory and invasive potentials of colon cancer. To identify whether *NEAT1*/miR‐185‐5p/*IGF2* axis participated in the progression of colon cancer, *NEAT1* and miR‐185‐5p were co‐overexpressed in HT‐29 cells. Overexpressed miR‐185‐5p downregulated *IGF2* expression in HT‐29 cells, but was further upregulated by co‐overexpressed *NEAT1* and miR‐185‐5p (Figure 5b). Overexpressed *NEAT1* partially reversed the inhibited migration and invasion of HT‐29 cells (Figure 5c). Conversely, cotransfection of miR‐185‐5p inhibitor and si‐*NEAT1* inhibited upregulated *IGF2* expression in SW480 cells with miR‐185‐5p knockdown (Figure 5d). *NEAT1* knockdown partially reversed the enhanced migration and invasion of SW480 cells (Figure 5e). It was concluded that the regulatory role of *NEAT1* in colon cancer depended on miR‐185‐5p/*IGF2*. In conclusion, this study revealed that the migration and invasion of colon cancer were regulated by *NEAT1*/miR‐185‐5p/*IGF2* axis (Figure 6).

**Figure 5:** *NEAT1*/MiR‐185‐5p axis was important in migratory and invasive potentials of colon cancer. (a) Invasive and migratory potentials were promoted by HT‐29 cells transfected with pcDNA‐*IGF2*, whereas the contrary trends were observed in SW480 cells transfected with si‐*IGF2*. (b) Overexpressed miR‐185‐5p downregulated *IGF2* expression in HT‐29 cells, but was further upregulated by co‐overexpressed *NEAT1* and miR‐185‐5p. (c) Overexpressed *NEAT1* partially reversed the migration and invasion of HT‐29 cells suppressed by miR‐185‐5p mimics. (d) Cotransfection of miR‐185‐5p inhibitor and si‐*NEAT1* suppressed the upregulated *IGF2* expression in SW480 cells with miR‐185‐5p knockdown. (e) *NEAT1* knockdown partially reversed the migration and invasion of SW480 cells promoted by miR‐185‐5p inhibitor. *p < .05

**Figure 6:** Summary of the regulation and mechanism of *NEAT1* in colon cancer

## 4 DISCUSSION

Several lncRNAs have been shown to participate in the progression of colon cancer. For instance, long noncoding RNA HNF1A‐AS1 mediated repression of miR‐34a/SIRT1/p53 feedback loop acts as a ceRNA to contribute to the metabolism of colon cancer (Fang et al., 2017). LncRNA BCAR4 contributes to the progression of colon cancer through the activation of Wnt/β‐catenin signaling (Ouyang et al., 2017). LncRNA MALAT1 induces the development of colon cancer through the regulation of miR‐129‐5p/HMGB1 axis (Wu, Meng, Jie, & Zhao, 2018). In this study, colon cancer patients presented with a high *NEAT1* expression relative to the controls. Moreover, the survival of colon cancer patients at a high *NEAT1* expression was shorter than those at low level. Overexpressed *NEAT1* considerably promoted migratory and invasive rates of colon cancer cells. Based on a series of functional analyses, *NEAT1* could mediate the progression of colon cancer through regulating *IGF2* by absorbing miR‐185‐5p.

RETRACTED

CeRNA hypothesis was proposed in 2011 for the first time (Giza, Vasilescu, & Calin, 2014). Moreover, lncRNAs shows interaction with target miRNA and further regulation of the expression of the target gene as ceRNAs together with direct gene expression regulation (Peng et al., 2016). CeRNA hypothesis is of crucial significance in regulating malignancies. In theory, all RNAs with miRNA‐binding sites could bind to miRNAs, followed by playing their roles as a ceRNA (Karreth & Pandolfi, 2013; Li, Sun, Hicks, & Raikhel, 2015). LncRNA/miRNA/mRNA network under ceRNA regulatory mode complements the miRNA function. This study revealed that the biological role of *NEAT1* in colon cancer depended on absorbing miR‐185‐5p. Bioinformatics prediction identified *IGF2* as a potential target gene of miR‐185‐5. *NEAT1* showed positive regulation on *IGF2* expression, whereas miR‐185‐5p showed negative regulation on it.

The expression of insulin‐like growth factor 2 (*IGF2*) is observed in the liver and many other tissues as a 7.5 kDa mitogenic peptide hormone (Livingstone, 2013). Overexpressed *IGF2* is observed in many cancers and is associated with a poor prognosis (Xu et al., 2017). The risk of various cancers (e.g., prostate, breast, ovarian) also increases with higher serum *IGF2* (Dong et al., 2015; Schagdarsurengin et al., 2017; Tominaga et al., 2017). This study showed a high expression of *IGF2* in colon cancer cells and tissues. Overexpressed *IGF2* contributed to invasive and migratory rates of colon cancer cells. It was more important that overexpressed *NEAT1* reversed the decrease in *IGF2* caused by miR‐185‐5p mimics, further suggesting that *IGF2* was a key target for *NEAT1* and miR‐185‐5p.

This research has several deficiencies. First, a larger sample size is required to further explore the clinical value of *NEAT1*. Second, which RNA domain of *NEAT1* long isoform comes in the contact with miR‐185‐3p needs further study. Third, more target genes or miRNAs should be applied to interact with *NEAT1*.

RETRACTED

This paper had some noteworthy limitations. This study placed emphasis on the in vitro roles of lncRNA *NEAT1*/miR‐185‐5p/*IGF2* axis in the progression of colon cancer. More experiments are warranted to confirm the effects of lncRNA *NEAT1*/miR‐185‐5p/*IGF2* on development and metastasis of colon cancer in vivo.

## 5 CONCLUSION

High *NEAT1* expression is observed in colon cancer, which contributes to the migration and invasion of colon cancer cells through absorbing miR‐185‐5p to upregulate *IGF2* expression. *NEAT1* is identified as an independent risk factor for poor prognosis of colon cancer.

## CONFLICT OF INTEREST

All authors declare no conflict of interest.
